This article has been retracted.

# Effects of Routine Health Care Combined with Oral Vitamin D on Linear Growth in 5-Year-Old Children

**DOI:** 10.1155/2022/4677795

**Published:** 2022-06-21

**Authors:** Qingwen Zeng, Yangyang Liu

**Affiliations:** ^1^Children Healthcare Center of Shiyan Maternal and Child Health Care Hospital, Shiyan, China; ^2^Children Rehabilitation Department of Shiyan Maternal and Child Health Care Hospital, Shiyan, China

## Abstract

**Objective:**

The aim is to evaluate the effects of routine health care combined with oral vitamin D on linear growth in 5-year-old children.

**Materials and Methods:**

The 5-year-old children who received routine health care in Shiyan Maternal and Child Health Care Hospital from January 2019 to January 2021 were retrospectively analyzed. They were divided into the supplement group and the non-supplement group according to whether or not they received oral vitamin D, and reasons for not taking oral vitamin D and its influence on children's linear growth were analyzed.

**Results:**

A total of 368 children were enrolled, including 228 children in the supplement group, accounting for 61.96%. The analysis of the influencing factors of vitamin D supplementation showed that the proportion of children with well-educated parents and living in cities and towns was higher (all *P* < 0.05). Comparing the general situation of children in the two groups, it was found that the height, weight, and head circumference of children in the supplement group were notably higher than those in the non-supplement group (all *P* < 0.05). At age 4 and 5, the height of the supplement group was significantly higher than that of the non-supplement group (all *P* < 0.001). Linear analysis showed that the relationship between height and age in the supplement group was *Y* (height, cm) = 10.07 × *X* (age, years) + 61.18, while that in the non-supplement group was *Y* (height, cm) = 8.296 × *X* (age, years) + 62.81, with significant difference (all *P* < 0.05). Serum 25-hydroxyvitamin D concentration in the supplement group was significantly higher than that in the non-supplement group, and the proportion of children ≥75 nmol/L was evidently higher than that in the supplement group (all *P* < 0.05). In addition, the incidence of vitamin D-related hypercalcemia in the supplement group was significantly higher than that in the non-supplement group (all *P* < 0.05).

**Conclusion:**

There are still more children without vitamin D supplement, which is closely related to their parents' education background and place of residence. Additionally, vitamin D supplementation can promote growth and improve 25-hydroxyvitamin D levels in children, but with the risk of related complications.

## 1. Introduction

Vitamin D is a steroid hormone that can promote the absorption of calcium and phosphorus by small intestinal mucosal cells, plays an important role in maintaining the calcium homeostasis of bone health, and functionally prevents the occurrence of rickets [1, 2]. After exposure to solar ultraviolet-B (UV-B) radiation, vitamin D can be synthesized naturally in the skin [3]. However, for any baby or child, the amount of sunlight required to prevent vitamin D deficiency is difficult to determine, and it is largely affected by the environment, including weather conditions, air pollution, caregiver habits, and the latitude where they live [4]. In addition, excessive intake of vitamin D can produce hypercalcemia, causing adverse reactions, such as dysuria, abdominal pain, and kidney stones, which seriously affect children's health [5, 6]. Linear growth retardation and developmental delay remain common indicators of malnutrition in children under 5 years of age and infants worldwide and are closely related to vitamin D deficiency [7, 8]. However, studies on the effects of vitamin D supplementation on linear growth and other health outcomes in infants and children under 5 years of age are scant. Our hospital intends to analyze the relationship between oral vitamins and linear growth in routine health care for children, and the reports are as follows.

## 2. Materials and Methods

### 2.1. General Information

Children under 5 years of age who underwent routine health care in Shiyan Maternal and Child Health Care Hospital from January 2019 to January 2021 were retrospectively analyzed, and informed consent has been obtained from all children guardians. Inclusion criteria were as follows: (1) children with age <5 years; (2) patients with full-term birth and breast feeding; (3) patients who establish a file for routine health care in this hospital, and have complete medical records; (4) parents or other guardians have normal communication skills. Exclusion criteria were as follows: (1) patients with multipl pregnancies; (2) patients combined with congenital genetic metabolic disease or infectious diseases; (3) patients with intrauterine growth restriction or combined with congenital growth and development defects; (4) patients combined with other important organ dysfunctions; (5) the patient's contraindications to the use of vitamin D; (6) patients who cannot cooperate to complete the inspection. The studies involving human participants were reviewed and approved by the Shiyan Maternal and Child Health Care Hospital, No. 29777-1.

### 2.2. Methods

All enrollments received regular health check-ups to monitor the baby's growth, exercise, and diet guidance. According to the use of vitamin D supplements when patients were enrolled, children were divided into the supplement group (daily oral vitamin D > 200 IU) and the non-supplement group (did not regularly supplement vitamins or did not meet the target). A self-made questionnaire was used to collect children's general information, birth information, family status, etc., to analyze the reasons for not supplementing vitamin D, and to compare the growth and development of the two groups of children.

### 2.3. Judgment Criteria

Children's fasting venous blood was collected, and radioimmunoassay was used to determine serum 25(OH)D concentration. Serum 25(OH)D < 25 nmol/L is considered lack of vitamin D; 25 nmol/L ≤ serum 25(OH)D < 75 nmol/L is defined as vitamin D deficiency; serum 25(OH)D ≥ 75 nmol/L means vitamin D is deemed as normal.

### 2.4. Statistical Methods

All data were analyzed by SPSS 23.0, and the GraphPad Prism 8.0 software was used to plot graphics. Measurement data were expressed as mean ± standard deviation, and two independent sample *t*-tests were employed for comparison between groups, and paired-sample *t*-tests for comparison within groups at different times; count data were expressed by rate, and examined by the chi-square test. The statistical difference was declared at *P* < 0.05.

## 3. Results

### 3.1. Analysis of Factors Affecting Vitamin D Supplementation

As shown in Table 1, all children were grouped according to whether they were supplemented with vitamin D. Among them, 228 children were supplemented with vitamin D, accounting for 61.96%. Comparing the basic information and family data of the two groups of children, it was found that the parent's educational background and place of residence were closely related to vitamin D supplementation. Children with highly educated parents and children living in cities and towns had a higher proportion of vitamin D supplementation (all *P* < 0.05), while gender, breastfeeding, gestational age, birth weight, etc., had no correlation with vitamin D supplementation (*P* > 0.05).

### 3.2. Comparison of Serum 25-Hydroxyvitamin D Levels between the Two Groups of Children

As shown in Table 2, the serum 25-hydroxyvitamin D level of the supplement group was noticeably higher than that of the non-supplement group, and the normal rate of 25-hydroxyvitamin D was considerably higher than that of the non-supplement group (*P* < 0.05).

### 3.3. Comparison of the Physical Development between the Two Groups of Children

As shown in Table 3, remarkably better the height, weight, and head circumference of the supplement group than the non-supplement group were observed (*P* < 0.001).

### 3.4. Comparison of Linear Growth between Two Groups of Children

As shown in Figures 1(a) and 1(b), there was no significant difference in height between the two groups at birth, 1 year old, 2 years old, and 3 years old (all *P* > 0.05); at 4 and 5 years old, the height of the supplement group was significantly higher than that of the non-supplement group (*P* < 0.001). Linear analysis showed that the relationship between height and age in the supplement group is *Y* (height, cm) = 10.07 × *X* (age, years) + 61.18, and the relationship between height and age in the non-supplement group is *Y* (height, cm) = 8.296 × *X* (age, years) + 62.81, the correlations were all significant (*P* < 0.05).

### 3.5. Comparison of the Incidence of Vitamin D-Related Adverse Reactions between the Two Groups of Children

As shown in Table 4, drastically higher proportion of elevated blood calcium was witnessed in the supplement group as compared with the non-supplement group (*P* < 0.05); the proportion of children with elevated urinary calcium and elevated plasma phosphate was not statistically different in the two groups (*P* > 0.05).

### 3.6. Comparison of Abnormal Growth and Development between the Two Groups of Children

As shown in Table 5, the proportion of low body weight in the supplement group was significantly lower than that in the non-supplement group (*P* < 0.05), and no notable disparity was found in the proportion of children with high body weight and neurobehavioral development delay between the two groups (*P* > 0.05).

## 4. Discussion

It is estimated that roughly one billion people in the world lacks vitamin D. Even in countries with whole-year sunshine, low vitamin D levels are a public concern faced by people of all ages [9, 10]. Children and infants are high-risk populations of vitamin D deficiency, which is attributed to insufficient outdoor activities, picky eaters, anorexia, etc.; additionally, rapid growth demands for vitamin D, which is likely to cause vitamin D deficiency [11, 12]. With the improvement of living conditions and the enhancement of health awareness, children health care has won popular support, and the harm of vitamin D deficiency has been widely recognized. However, 38.04% of children under routine health care in this study still have no regular vitamin D supplementation. Children under 3-year-old are the target for vitamin D supplementation and rickets prevention and treatment, as a result, older children are less regularly supplemented with vitamin D preparations, and most natural foods contain low vitamin D content, leading to insufficient intake [13]. Moreover, this study found that the parents' education background and place of residence are closely related to vitamin supplementation. Parents are the main caregivers of children. Parents with higher educational background have richer knowledge of scientific parenting and pay more attention to the children's nutrition and health; children living in cities and towns enjoy better medical conditions, and more extensive propaganda and education about vitamin D supplementation [14, 15].

In this study, it is shown that high school-aged children are prone to insufficient vitamin D production due to increased academic burden, reduced outdoor activities, and sunshine time. 25(OH)D is an indicator to evaluate the body's vitamin D status, but the threshold value between shortage and deficiency remains controversial [16]. It is generally considered that serum 25(OH)D < 25 nmol/L is lack of vitamin D; 25 nmol/L ≤ serum 25(OH)D < 75 nmol/L indicates vitamin D deficiency; serum 25(OH)D ≥ 75 nmol/L indicates normal vitamin D. In this study, the normal rate of children without vitamin D supplementation was 60.00%, indicating that the amount of vitamin D produced by simple diet and sunlight exposure is very low, and oral vitamin D supplementation is necessary.

Linear growth disorder plays a negative role in the children's health and neurodevelopmental status, and is also related to school performance and work ability decline, physical decline, chronic disease, or poor cognitive ability in adulthood [17]. Linear growth retardation is triggered by many factors, including shortness of the mother, intrauterine growth restriction, premature infants, low birth weight infants, and malnutrition. In addition, repeated infections, environmental enteropathy, and insufficient care are all contributed to linear growth disorders [18, 19]. In this study, the relationship between the height and age in the supplement group was *Y* (height, cm) = 10.07 × *X* (age, years) + 61.18, and the relationship between height and age in the non-supplement group was *Y* (height, cm) = 8.296 × *X* (age, years) + 62.81, the correlations bear significance. Vitamin D plays a crucial role in maintaining bone health. It regulates calcium and phosphorus metabolism together with parathyroid hormone and calcitonin, and it promotes bone growth, which is consistent with the results of this study [20]. Insufficient vitamin D can impede the healthy development of the bone and extra-skeletal, but there is a controversy about the relationship between the children's linear growth and vitamin D.

Studies have shown that high-dose vitamin D supplementation may have a negative impact on the linear growth of children, by comparing the development of infants with a daily intake of more than 1500 UI of vitamin D and 300–600 UI, and found that the growth rate of infants in the high-dose group was reduced [21]. Previous studies pointed out that oral vitamins generate slight influence on children's linear growth, growth retardation, hypercalcemia, etc., only yield a light increase in the linear growth index of low-birth-weight infants. A prior trail stated that 2000 UI of vitamin D supplementation per day during infancy has little connection with height loss at any age [22]. Therefore, the relationship between vitamin D and linear growth needs to be confirmed by further studies, which may be closely related to the intake dose. Inevitably, limitations should also be highlighted albeit the reference value it provides. The sample in the current study was selected from a certain region of China. Hence, findings should be interpreted with cautions due to its restricted universality. Medical technology and the continuous improvement of the people's quality of life, children's health care, and gradually more attention to the development trend of diversification. Traditional Chinese medicine health care intervention in the development of children is obtaining more and more staff attention.

## 5. Conclusion

There are still more children without vitamin D supplementation, which is closely related to their parents' education and place of residence. Additionally, vitamin D supplementation can promote the growth and development of children, and improve the level of 25(OH)D, yet with an odd of related complications.

## Figures and Tables

**Figure 1:** The linear relationship between age and height.: (a) The supplement group and (b) the non-supplement group.

**Table 1:** Analysis of factors affecting vitamin D supplementation.

	Supplement group (*n* = 228)	Non-supplement group (*n* = 140)	*t*/*χ*^2^	*P*
Gender			0.561	0.454
Male	146	95		
Female	82	45		
Breast feeding			1.291	0.256
Yes	196	126		
No	32	14		
Embryonic days	38.68 ± 2.55	39.12 ± 2.95	1.513	0.131
Birth weight	3.58 ± 0.92	3.64 ± 1.12	0.558	0.577
Parents' education level			9.436	0.002
Junior college or below	88	77		
Bachelor degree or above	140	63		
Residence			4.499	0.034
Rural	42	39		
Cities and towns	186	101		

**Table 2:** Comparison of the physical development between the two groups of children.

	Height	Body weight	Head girth
Supplement group (*n* = 228)	107.07 ± 13.58	24.95 ± 6.28	57.68 ± 6.11
Non-supplement group (*n* = 140)	99.25 ± 12.25	20.48 ± 5.95	54.24 ± 5.76
*t*	5.563	6.762	5.358
*P*	<0.001	<0.001	<0.001

**Table 3:** Comparison of serum 25-hydroxyvitamin D levels between the two groups of children.

	Lack of vitamin D	Vitamin D deficiency	Normal vitamin D
Supplement group (*n* = 228)	1	22	205 (89.91)
Non-supplement group (*n* = 140)	13	43	84 (60.00)
*t*/*χ*^2^			46.03
*P*			<0.001

**Table 4:** Comparison of the incidence of vitamin D-related adverse reactions between the two groups of children.

	Elevated urinary calcium	Elevated blood calcium	Elevated plasma phosphate
Supplement group (*n* = 228)	35	44	42
Non-supplement group (*n* = 140)	12	14	16
*χ* ^2^	3.578	5.648	3.194
*P*	0.059	0.017	0.074

**Table 5:** Comparison of abnormal growth and development between the two groups of children.

	Low body mass	High body mass	Neurobehavioral developmental delay
Non-supplement group (*n* = 140)	16 (11.43)	18 (12.86)	14 (10.00)
Supplement group (*n* = 228)	12 (5.26)	44 (19.30)	19 (8.33)
*χ* ^2^	4.69	2.569	0.295
*P*	0.030	0.109	0.587

## Data Availability

The data used to support the findings of this study are available from the corresponding author upon request.
